The article "miR-663 attenuates tumor growth and invasiveness by targeting eEF1A2 in pancreatic cancer" was retracted in 2019. Reasons: duplicated images; overlap with earlier publications; unreliable data.

# miR-663 attenuates tumor growth and invasiveness by targeting eEF1A2 in pancreatic cancer

**DOI:** 10.1186/s12943-015-0315-3

**Published:** 2015-02-13

**Authors:** Wenqiao Zang, Yuanyuan Wang, Tao Wang, Yuwen Du, Xiaonan Chen, Min Li, Guoqiang Zhao

**Affiliations:** College of Basic Medical Sciences, Zhengzhou University, Zhengzhou, 450001 Henan Province China; Department of Hemato-tumor, The First Affiliated Hospital of Henan University of TCM, Zhengzhou, 450000 China

**Keywords:** miR-663, Growth, Invasion, eEF1A2, Pancreatic cancer

## Abstract

**Background:**

miR-663 is associated with many important biologic processes, such as the evolution, development, viral infection, inflammatory response, and carcinogenesis among vertebrates. However, the molecular function and mechanism of miR-663 in pancreatic cancer growth and invasion is still unclear.

**Methods:**

Western blot and real-time PCR were used to study the expression level of eEF1A2 protein and miR-663 in pancreatic cancer tissues and cell lines. The Pearson *χ*^2^ test was used to determine the correlation between miR-663 expression and clinicopathologic features of patients. Patients’ survival was analyzed using the Kaplan–Meier method, using the log-rank test for comparison. The biological function of miR-663 was examined by measuring cell growth, cell invasion and apoptosis analysis in vitro and in vivo. miR-663 target gene and signaling pathway was identified by luciferase activity assay and western blot.

**Results:**

We found that, in pancreatic cancer, eEF1A2 was significantly upregulated but miR-663 was significantly downregulated. Further results showed that the expression level of eEF1A2 and miR-663 was strongly associated with TNM stage and node metastasis status of the patients. miR-663 and eEF1A2 were inversely correlated with each other, and the changes in the expression levels of each can also predict the survival of patients with pancreatic cancer. We identified miR-663 as a tumor attenuate molecular that attenuated the proliferation and invasion of pancreatic cancer cells both in vitro and in vivo. Finally, we confirmed that the expression of eEF1A2 can partially restore the pro-apoptotic and anti-invasion functions of miR-663.

**Conclusions:**

miR-663 attenuated the proliferation and invasion of pancreatic cells both in vitro and in vivo by directly targeting eEF1A2. miR-663 and eEF1A2 might be potential targets for the treatment of pancreatic cancer in the future.

## Background

Pancreatic cancer is one of the poorest prognoses among human tumors, with an overall 5-year survival rate of less than 5% [1]. In spite of the continuous developments in clinical therapies and novel surgical techniques, the survival of patients with pancreatic cancer has remained poor for over 30 years [2]. Pancreatic cancer is highly aggressive, wherein tissue invasion and remote metastasis may occur during the early stages [3]. Because invasion and metastasis are the most formidable obstacles preventing the effective treatment of pancreatic cancer, it is therefore essential to explore the molecular mechanisms that contribute to this aggressive behavior, in order to improve the outcomes for patients.

miR-663, a member of the primate-specific miRNA family, is associated with many important biologic processes, including the evolution, development, viral infection, inflammatory responses, and carcinogenesis of many vertebrate species [4-9]. However, its role in tumor progression can be considered quite contradictory. Although it acts as an oncogene that promotes the malignancy of lung cancer, nasopharyngeal carcinoma, and breast cancer [6,7], miR-663 may also act as a potential tumor attenuate molecular in gastric cancer, colorectal carcinoma, prostate cancer, and acute lymphoblastic leukemia [8,9]. Overall speaking, the effect and mechanism of miR-663 on pancreatic cancer remain unclear.

Eukaryotic elongation factor 1-a (eEF1A) is a member of the G protein family, and one of the four subunits that constitute the eukaryotic elongation factor 1 [10,11]. And it has two identified isoforms, namely eEF1A1 and eEF1A2. Unlike eEF1A1, which is expressed almost ubiquitously, eEF1A2 is normally only present in the heart, brain, and skeletal muscles [12-14]. eEF1A2 is involved in a variety of biological processes such as cytoskeleton modification [13,14], targeting proteins for degradation [15], heat shock response [16], apoptosis [17], and phosphatidylinositol signaling [18,19]. eEF1A2 is considered as an oncogene marker because it is highly expressed in a subset of cancers, such as ovarian cancer [20], breast cancer [21], and pancreatic cancer [22].

In the present study, we evaluated the expression and clinical relevance of miR-663 and eEF1A2 in pancreatic cancer. Additionally, we investigated the functional role of miR-663 in the invasion of pancreatic cancer cell lines. The contribution of miR-663 to pancreatic cancer malignancy and the underlying molecular mechanisms were also investigated. Our data demonstrate that miR-663 has potential value as a prognostic marker and as a therapeutic target of pancreatic cancer.

## Results

### eEF1A2 is upregulated and miR-663 is downregulated in pancreatic cancer

Western blot and real-time PCR were used to study the expression level of eEF1A2 protein and miR-663 in pancreatic cancer tissues. To analyze the clinicopathological significance of eEF1A2 and miR-663, we examined 68 primary pancreatic cancer tissues, as well as 68 normal pancreas tissues, collected from sites adjacent to tumors. The relationship between the expression level of eEF1A2 and miR-663, and the clinicopathologic characteristics in pancreatic cancer patients were summarized in Table 1. Compared with normal pancreatic tissues adjacent to tumors, the expression level of eEF1A2 protein was generally upregulated in pancreatic cancer tissues (Figure 1A, B). On the contrary, the average expression level of miR-663 was decreased in pancreatic cancer tissue (Figure 1C).

**Table 1:** **Clinicopathological characteristics of pancreatic cancer patients**

**Parameter**		**eEF1A2 protein**		**miR-663**	
		**Expression level**	**P value**	**Expression level**	**P value**
Gender					
Male	45	0.706 ± 0.1486	0.230	0.421 ± 0.2493	0.426
Female	23	0.750 ± 0.1272		0.374 ± 0.1669	
Age (years)					
<60	42	0.702 ± 0.1515	0.163	0.422 ± 0.2552	0.436
≥60	26	0.751 ± 0.1227		0.378 ± 0.1649	
Diameter (cm)					
<3	51	0.715 ± 0.1471	0.566	0.425 ± 0.2322	0.218
≥3	17	0.738 ± 0.1294		0.347 ± 0.1947	
Location					
Head	48	0.713 ± 0.1394	0.486	0.398 ± 0.2057	0.663
Body, tail	20	0.739 ± 0.1511		0.423 ± 0.2696	
Differentiation					
Well	13	0.643 ± 0.1667		0.518 ± 0.3358	
Moderate	39	0.735 ± 0.1265	0.086	0.383 ± 0.1812	0.124
Poor	16	0.747 ± 0.1453		0.366 ± 0.1947	
TNM stage					
I-II	30	0.670 ± 0.1635	0.009*	0.498 ± 0.2742	0.004*
III-IV	38	0.760 ± 0.1098		0.332 ± 0.1411	
Nodal status					
Negative	36	0.688 ± 0.1632	0.048*	0.464 ± 0.2623	0.017*
Positive	32	0.757 ± 0.1057		0.338 ± 0.1505	

*Indicated statistical significance (*P* < 0.05).

**Figure 1:** **The expression levels of eEF1A2 protein and miR-663 in pancreatic cancer tissues and cell lines. A**. The expression levels of eEF1A2 protein in paired pancreatic cancer tissues and adjacent non-tumor tissues. **B**. eEF1A2 protein expression level in pancreatic cancer tissues was higher than in adjacent non-cancerous tissues. **C**. miR-663 expression level in pancreatic cancer tissues was lower than in adjacent non-cancerous tissues. **D**. eEF1A2 protein expression levels in TNM stage I-II were lower than in TNM stage III-IV in pancreatic cancer tissues. **E**. eEF1A2 protein expression levels in pancreatic cancer tissues with positive node metastasis were higher than with negative node metastasis. **F**. miR-663 expression levels in TNM stageI-II were higher than in TNM stage III-IV in pancreatic cancer tissues. **G**. miR-663 expression levels in pancreatic cancer tissues with positive node metastasis were lower than with negative node metastasis. **H**. eEF1A2 protein expression level in pancreatic cancer cell lines were higher than in the normal pancreatic cell line. **I**. miR-663 expression level in pancreatic cancer cell lines were lower than in the normal pancreatic cell line. **J**. eEF1A2 and miR-663 have an inverse correlation.

The further results showed that eEF1A2 and miR-663 expression level were strongly associated with the TNM stage and nodal status of the patients, not associated with age, gender, diameter, location and differentiation (Table 1). We found that eEF1A2 expression was lower in stage I-II, but higher in stages III-IV; this reflects that eEF1A2 has a significant correlation with clinical stages (Figure 1D, Table 1). But the expression of miR-663 was higher in stage I-II, whereas it is lower in stages III-IV, this reflects that miR-663 has a significant correlation with clinical stages (Figure 1F, Table 1). In addition, we found that the level of eEF1A2 was higher in the presence of lymph node metastasis than in the absence of lymph node metastasis (Figure 1E, Table 1). The expression level of eEF1A2 exhibits a different pattern from miR-663 (Figure 1G, Table 1). The level of miR-663 was lower with lymph node metastasis than without (Figure 1G, Table 1). Taken together, these data provided strong evidence that the miR-663 expression was closely related to the progression and clinicopathologic features of pancreatic cancer. We further tested the expression level of eEF1A2 and miR-663 in pancreatic cancer cell lines to analyze their clinicopathological significance. Consistent with the result of the pancreatic cancer tissues, compared with the normal pancreatic cell line PDE6-C7, the expression level of eEF1A2 protein was generally upregulated in pancreatic cancer cell lines (PANC-1, Capan-2, SW1990, BxPC3 and AsPC-1) (Figure 1H). On the contrary, the basal expression level of miR-663 was generally downregulated in pancreatic cancer cell lines (PANC-1, Capan-2, SW1990, BxPC3 and AsPC-1) (Figure 1I). On the basis of these results, we focused on miR-663 for further functional studies on its roles in pancreatic cancer pathogenesis.

To investigate the correlation between miR-663 and eEF1A2, we examined their expressions in primary human pancreatic cancer tissues. Unlike the matched normal pancreatic tissues, in the tumor tissues from the 68 patients with pancreatic cancer, miR-663 was reduced, whereas eEF1A2 protein was increased, which demonstrates a significant negative correlation (R^2^ = 0.624; *P* < 0.01; Figure 1J). The data suggested that eEF1A2 and miR-663 have an inverse correlation in pancreatic cancer tissues.

### eEF1A2 and miR-663 are associated with the survival of patient in pancreatic cancer

We used Kaplan-Meier method to analyze the relationship between clinicopathologic characteristics and patient survival rates, based on follow-up visits of pancreatic cancer patients. The results showed that tumor diameter (*P* < 0.001; Figure 2A), differentiation (*P* < 0.001; Figure 2B), clinical stage (*P* < 0.001; Figure 2C) and lymph node metastasis (*P* < 0.001; Figure 2G) were all significantly associated with the survival of patients. But the gender (*P* = 0.975; Figure 2D), age (*P* = 0.523; Figure 2E) and location (*P* = 0.613; Figure 2F) were not significantly associated with the survival of patients.

**Figure 2:** **The survival of patient in pancreatic cancer.** Patients’ survival was analyzed using the Kaplan–Meier method, with the log-rank test for comparison. A statistically significant difference (*P* < 0.05) was observed. **A**. Tumor diameter was strongly associated with the survival of patients. **B**. Differentiation was significantly associated with the survival of patients. **C**. The clinical stage was significantly associated with the survival of patients. **D**. Gender was not significantly associated with the survival of patients. **E**. Age was not significantly associated with the survival of patients. **F**. Location was not significantly associated with the survival of patients. **G**. Lymph node metastasis was significantly associated with the survival of patients. **H**. eEF1A2 expression was significantly associated with the survival of patients. **I**. miR-663 expression was significantly associated with the survival of patients.

To validate the relationship between the expression of eEF1A2 and miR-663, and the survival of patient in pancreatic cancer, we examined the endogenous eEF1A2 and miR-663 expression in pancreatic cancer tissues, and we observed through the Kaplan-Meier analysis that the patients with higher level of eEF1A2 (≥0.72) had shorter survival (*P* < 0.001; Figure 2H). On the contrary, the patients with higher level of miR-663 (≥0.397) had longer survival (*P* < 0.001; Figure 2I). Taken together, the results above suggest that eEF1A2 and miR-663 are both associated with the survival of patient in pancreatic cancer. eEF1A2 and miR-663 may be potential biomarkers for prognosis in patients with pancreatic cancer.

### miR-663 attenuates pancreatic cancer cell proliferation

The frequent downregulation of miR-663 in both pancreatic cancer tissues and pancreatic cancer cell lines indicated that miR-663 might play a role in pancreatic cancer tumorigenesis. To explore the potential tumor attenuate effect of miR-663, we first synthesized a miR-663 agomir or a miR-663 scramble, and then transfected PANC-1 and AsPC-1 cells with them. The upregulated expression of miR-663 was confirmed by Real-time PCR (Figure 3A). CCK-8 and colony formation assays were utilized to evaluate cell proliferative capacity. As was shown in Figure 3B and C, after transfection for 24 h, 48 h and 72 h, the miR-663 group revealed a significant slower proliferation than the control groups (Blank and NC groups) for PANC-1 (Figure 3B) and AsPC-1 cells (Figure 3C). Consistent with the results of CCK8, The upregulated expression of miR-663 also visibly attenuated colony formation. The colony numbers of PANC-1(Figure 3D) and AsPC-1 cells (Figure 3E) were 62.3 ± 8.4 and 42.5 ± 5.7, respectively, in miR-663 group. These results suggested that miR-663 could attenuate the proliferation of pancreatic cancer cells in vitro, and might function as tumor attenuate molecular in vitro.

**Figure 3:** **miR-663 attenuates pancreatic cancer cell proliferation. A**. The expression of miR-663 was upregulated in the cells trasfected with miR-633 agomir. The expression of miR-663 was measured by RT-PCR. **B**. A statistically significant decrease in PANC-1 cell proliferation in the miR-663 group was observed compared to the Blank and NC groups. Effect of miR-663 on cell proliferation was measured by CCK-8 assay. **C**. A statistically significant decrease in AsPC-1 cell proliferation in the miR-663 group was observed compared to the Blank and NC groups. Effect of miR-663 on cell proliferation was measured by CCK-8 assay. **D**. miR-663 transfection of PANC-1 reduced growth of colonies. Colony formation in soft agar after 14 days using PANC-1 exposed to miR-663. Quantification of clone number per 10× microscopic field for cells exposed to miR-663 in duplicate experiments performed with triplicate wells. Compared to the Blank and NC groups, a significant reduction (*P < 0.05) in colony forming potential was observed after treatment with miR-663 as assessed by counting the number of clones. **E**. miR-663 transfection of AsPC-1 reduced growth of colonies. Colony formation in soft agar after 14 days using AsPC-1 exposed to miR-663. Quantification of clone number per 10× microscopic field for cells exposed to miR-663 in duplicate experiments performed with triplicate wells. Compared to the Blank and NC groups, a significant reduction (*P < 0.05) in colony forming potential was observed after treatment with miR-663 as assessed by counting the number of clones.

### miR-663 attenuates pancreatic cancer cell invasiveness

We next tested whether miR-663 could alter the invasiveness of pancreatic cancer cells in vitro. To study the effect of miR-663 on the invasiveness of pancreatic cancer, PANC-1 and AsPC-1 cells were transfected with either miR-663 agomir (miR-663 group) or miR-663 scramble using a Matrigel model (NC group). In vitro, more specifically in the PANC-1 (18.4 ± 3.2, *P* < 0.01, Figure 4A) and AsPC-1 (15.7 ± 3.1, *P* < 0.01, Figure 4B) cells, pancreatic cancer’s invasive growth was significantly impaired when transfected with miR-663 agomir, as compared to the Blank and NC groups.

**Figure 4:** **miR-663 attenuates pancreatic cancer cell invasiveness. A**. miR-663 attenuates pancreatic cancer PANC-1 cell invasiveness. Invasive ability of PANC-1 after transfection was assessed using Transwell assays. The number of invasive miR-663-transfected PANC-1 cells was significantly lower than in the Blank and NC groups. *P < 0.05 compared to the control group. **B**. miR-663 attenuates pancreatic cancer AsPC-1 cell invasiveness. Invasive ability of AsPC-1 after transfection was assessed using transwell assays. The number of invasive miR-663-transfected AsPC-1cells was significantly lower than in the Blank and NC groups. *P < 0.05 compared to the control group. **C**. miR-663 attenuates protein expression of MMP9, Akt, pAkt and eEF1A2 in PANC-1 cells. Protein expression was measured by Western blot assay. miR-663 significantly attenuates protein expression of MMP9 , Akt and pAkt in PANC-1 cells compared to the Blank and NC groups. β-actin was used as a reference. **D**. miR-663 attenuates protein expression of MMP9, Akt, pAkt and eEF1A2 in AsPC-1 cells. Protein expression was measured by Western blot assay. miR-663 significantly attenuates protein expression of MMP9, Akt and pAkt in AsPC-1 cells compared to the Blank and NC groups. β-actin was used as a reference.

The matrix metalloproteinases (MMPs) are family members of extracellular proteinases that regulate basic cellular processes including survival, migration, morphogenesis and degradation of extracellular matrix during the cancer metastatic process [23,24]. Among the MMPs members, MMP9 cleaves the extracellular domain of NOTCH1 and activates NOTCH1 downstream target gene expression [25,26]. Akt, also known as protein kinase B (PKB), is a serine/threonine-specific protein kinase that plays a key role in multiple cellular processes such as glucose metabolism, apoptosis, cell proliferation, transcription and cell migration [27]. Once correctly positioned at the membrane via PIP3 binding, Akt can then be phosphorylated by its activating kinases. Akt regulates cellular survival and metabolism by binding and regulating many downstream effectors [28]. We examined the expression levels of MMP9, Akt and pAkt(Ser473), and found that the ectopic expression of miR-663 markedly attenuated the protein expression of MMP9, Akt and pAkt in both PANC-1 (Figure 4C) and AsPC-1 cells (Figure 4D), and is concomitant with the attenuation of cell invasion. These results suggest that miR-663 could attenuate pancreatic cancer cell invasiveness, which is likely associated with MMP9 and Akt.

### miR-663 induces cell apoptosis

To determine whether the decrease in pancreatic cancer growth by miR-663 was due to an induction of apoptosis, we evaluated the rate of cellular apoptosis using the FITC Annexin V Apoptosis Detection Kit I (BestBio, Shanghai, China) by flow cytometry. The results showed that the numbers of both early and late apoptotic cells at 48–96 h post-transfection of miR-663 agomir in PANC-1 (Figure 5A) and AsPC-1 cells (Figure 5B) significantly increased when compared to the miRNA transfected control group (NC group). Consistent with the results from the flow cytometry assay, the upregulated expression of miR-663 also noticeably induced apoptosis of PANC-1 (Figure 5C) and AsPC-1 cells (Figure 5D) in the Hoechst 33342 staining assay. The results suggest that miR-663 induces cell apoptosis.

**Figure 5:** **miR-663 induces cell apoptosis in PANC-1 and AsPC-1 cells. A**. miR-663 induces PANC-1cell apoptosis. The apoptosis cells of PANC-1 were assessed using flow cytometry assay. The number of apoptosis miR-663-transfected PANC-1 cells was significantly higher than in the Blank and NC groups. *P < 0.05 compared to the control group. **B**. miR-663 induces AsPC-1 cell apoptosis. The apoptosis cells of AsPC-1 were assessed using flow cytometry assay. The number of apoptosis miR-663-transfected AsPC-1 cells was significantly higher than in the Blank and NC groups. *P < 0.05 compared to the control group. **C**. Results from Hoechst 33342 staining assay showed that transfection with the miR-663 agomir led to a significant increase in PANC-1 cell apoptosis compared to the Blank and NC groups (*P* < 0.05). **D**. Results from Hoechst 33342 staining assay showed that transfection with the miR-663 agomir led to a significant increase in AsPC-1 cell apoptosis compared to the Blank and NC groups (*P* < 0.05). **E**. miR-663 increased protein expression of BAD, BAX, and cleaved caspase-3 in PANC-1 cells. Protein expression was measured by Western blot assay. The protein levels of BAD, BAX and cleaved caspase-3 were enhanced in miR-663 group in PANC-1 cells compared to the Blank and NC groups. β-actin was used as a reference. **F**. miR-663 increased protein expression of BAD, BAX and cleaved caspase-3 in AsPC-1 cells. Protein expression was measured by Western blot assay. The protein levels of BAD, BAX and cleaved caspase-3 were enhanced in miR-663 group in AsPC-1 cells compared to the Blank and NC groups. β-actin was used as a reference.

BAD, a protein related to Bcl-2, is a promoter of apoptosis, which has been shown to dimerize with anti-apoptotic proteins Bcl-2 and Bcl-XL. BAD connects the upstream signal transduction paths with the BCL-2 family, and modulate this checkpoint for apoptosis [29]. BAX, a death-promoting member critical to cell death, heterodimerizes with multiple death-repressing molecules [30]. Induction of apoptosis was further confirmed by the expression of apoptosis related proteins using western blot. As shown in Figure 5E and F, the protein levels of BAD, BAX, and cleaved caspase-3 were enhanced in miR-663 group in PANC-1 and AsPC-1 cells compared to the Blank and NC groups. These results inferred that miR-663 induced cell apoptosis by regulating the BAD-dependent apoptosis pathway. The apoptosis must be contributing factors leading to the growth attenuation in pancreatic cancer cells that express miR-663.

### miR-663 attenuates tumor growth in vivo

To further confirm the growth-attenuating effect of miR-663 on pancreatic cancer, a xenograft tumor growth assay was performed. The subcutaneous tumor volume growth curve of PANC-1 stably expressed miR-663 or Blank control in vivo was shown in Figure 6A. The tumor volume was significantly lower in the miR-663 nude mice as compared to the control mice at 2, 3, 4 week. (*P* < 0.05, Figure 6A). After 4 weeks, the tumors were harvested (Figure 6B). The total weight of the metastatic tumors was significantly lower in miR-663 nude mice as compared to the control mice (Figure 6C). Our results revealed that miR-663 could attenuate the proliferation of pancreatic cancer cells in vivo. These results provide further evidence that miR-663 plays a tumor attenuated role in pancreatic cancer.

**Figure 6:** **MiR-663 inhibited tumor growth in vivo. A**. The subcutaneous tumor volume growth curve of PANC-1 stably expressed miR-663 or Blank control in vivo was shown. The tumor volume was significantly lower in miR-663 nude mice as compared to the control nude mice. **B**. Tumors were harvested after 4 weeks. **C**. The total weight of the metastatic tumors in each group. Significant difference (*P < 0.05).

### miR-663 targets eEF1A2 via binding to its 3’UTR

We searched for the direct target of miR-663 based on the following criteria: the target should have oncogenic property and should regulate cell migration and invasion. Among these targets of miR-663 predicted by the bioinformatics algorithms (TargetScan and miRBase), we focused on eEF1A2. The 3′ untranslated region (3′UTR) of eEF1A2 contains a seed region for miR-663 (Figure 7A). To test the specific regulation through the seed region, we constructed a reporter vector which consists of the luciferase coding sequence followed by the 3′UTR of eEF1A2. Either the wild type (pmirGLO-eEF1A2-3′UTR) or the mutated sequence (pmirGLO-eEF1A2-mut 3′UTR) within the seed region sites was cloned into the pmirGLO reporter vector (Figure 7A). Co-transfection experiments showed that miR-663 significantly decreased the luciferase activity of the wild type in PANC-1 (*P* < 0.05, Figure 7C) and AsPC-1 cells (*P* < 0.05, Figure 7D); but this was not observed in the mutant type (Figure 7C, D). Our data thus demonstrated that eEF1A2 was a direct target of miR-663.

**Figure 7:** **eEF1A2 is the direct target of miR-663 in PANC-1 and AsPC-1 cells. A**. The putative miR-663 binding sequences for the eEF1A2 3′ UTRs. The 3′ untranslated region (3′UTR) of eEF1A2 contains a seed region for miR-663. **B**. Western blot analysed eEF1A2 expression in transfected cells. Transfection of miR-663 agomir resulted in significant reduction of eEF1A2 protein expression by western blot in PANC-1 and AsPC-1 cells. β-actin was used as a reference. **C**. miR-663 significantly decreased the luciferase activity of wild type in PANC-1. **D**. miR-663 significantly decreased the luciferase activity of wild type in AsPC-1 cells. (*P < 0.05).

To further confirm that miR-663 targets eEF1A2, miR-663 agomir or miR-663 scramble was transfected into PANC-1 and AsPC-1 cells. Transfection of miR-663 agomir resulted in significant reduction of eEF1A2 protein expression by western blot in PANC-1 and AsPC-1 cells, respectively (*P* < 0.05, Figure 7B). These results show that miR-663 targets eEF1A2 by binding to its 3′UTR in pancreatic cancer cells.

### Expression of eEF1A2 could partially restore the pro-apoptotic function and anti- invasion of miR-663

To explore the function of eEF1A2 in pancreatic cancer cells, we constructed pcDNA3.1- eEF1A2 lacking the 3′ UTR, and we then transfected them into PANC-1 cells. Western blot assay showed that the transfection of miR-663 agomir inhibited the expression of eEF1A2 (Figure 8A). Co-transfection of pcDNA3.1-eEF1A2 and miR-663 abrogated the effects of miR-663 on eEF1A2 expression (Figure 8A). Our apoptosis assay indicated that the exogenous expression of miR-663 increased cell apoptosis that was induced by serum starvation (Figure 8B). Subsequently, we exogenously expressed the recombinant eEF1A2 lacking the 3′ UTR sequence (pcDNA3.1-eEF1A2) in PANC-1 cells. Cells transfected with pcDNA3.1-eEF1A2 alone showed significantly decreased levels of apoptosis (Figure 8B). However, when we co-transfected the cells with pcDNA3.1-eEF1A2 and miR-663, the expression of eEF1A2 lacking the 3′ UTR sequence was found to restore the pro-apoptotic functions of miR-663 (Figure 8B).

**Figure 8:** **Expression of eEF1A2 restored the pro-apoptotic function and anti-migration of miR-663. A**. eEF1A2 protein level was detected by western blot assay. Cells were transfected with pcDNA3.1- eEF1A2 (not including 3′UTR) or (and) miR-663. Western blot assay showed that transfection of miR-663 agomir inhibited the expression of eEF1A2. Co-transfection of pcDNA3.1- eEF1A2 and miR-663 abrogated the effects of miR-663 on eEF1A2 expression. β-actin was used as a reference. **B**. Expression of eEF1A2 restored the pro-apoptotic function of miR-663. Cells were transfected with pcDNA3.1- eEF1A2 (not including 3′ UTR) or (and) miR-663. The cell apoptosis were assessed using flow cytometry assay. Co-transfected cells with pcDNA3.1- eEF1A2 and miR-663, the expression of eEF1A2 lacking the 3′ UTR sequence was found to restore the pro-apoptotic functions of miR-663. **C**. Expression of eEF1A2 restored the anti-migration function of miR-663. Cells were transfected with pcDNA3.1- eEF1A2 (not including 3′ UTR) or (and) miR-663. Invasive ability was assessed using transwell assays. Co-transfected cells with pcDNA3.1- eEF1A2 and miR-663, the expression of eEF1A2 lacking the 3′ UTR sequence was found to restore the anti-migration functions of miR-663.

In the transwell assays we found that the exogenous expression of miR-663 decreased cell invasiveness (Figure 8C). Subsequently, we exogenously expressed the recombinant eEF1A2 lacking the 3′ UTR sequence (pcDNA3.1- eEF1A2) in PANC-1 cells. Cells transfected with pcDNA3.1- eEF1A2 alone showed significantly increased cell invasiveness (Figure 8C). But when the cells were co-transfected with pcDNA3.1- eEF1A2 and miR-663, the expression of eEF1A2 lacking the 3′ UTR sequence was found to restore the anti-invasion of miR-663 (Figure 8C). From these results we concluded that the expression of eEF1A2 could partially restore the pro-apoptotic function and anti-invasion of miR-663.

### eEF1A2 silencing and miR-663 overexpression exert anti-proliferative, anti-invasive and pro-apoptotic effects on pancreatic cancer cells

To further explore the biological significance of eEF1A2 and miR-663 in pancreatic cancer cells, eEF1A2-siRNAs and miR-663 agomir were transfected into PANC-1 cells. CCK8 array showed that the silencing of eEF1A2 and the overexpression of miR-663 attenuated cell proliferation (Figure 9A). This attenuation is more obvious in PANC-1 cells overexpressing miR-663. Furthermore, Colony formation assay obtained the same results—namely, that the silencing of eEF1A2 and the overexpression of miR-663 attenuated PANC-1 cells proliferation (Figure 9B). Invasion assay showed that the knockdown of eEF1A2 and the overexpression of miR-663 repressed the invasion and invasion capacities of PANC-1 cells (Figure 9C). For PANC-1 cells over-expressing miR-663, the invasion was more clearly attenuated (Figure 9C). To investigate the effect of eEF1A2-siRNAs and miR-663 on apoptosis, we performed apoptosis assay. As showed in Figure 9D, compared to the Blank control, eEF1A2 silencing and the overexpression of miR-663 significantly induced PANC-1 cell apoptosis.

**Figure 9:** **eEF1A2 silencing and miR-663 overexpression exert anti-proliferative, anti-invasive and pro-apoptotic effects on pancreatic cancer cells. A**. eEF1A2 silencing and miR-663 overexpression inhibited the proliferation. CCK8 array was used to assess PANC-1 proliferation. **B**. eEF1A2 silencing and miR-663 overexpression reduced growth of colonies of PANC-1 cells (*P < 0.05). Colony formation assay was used. **C**. eEF1A2 silencing and miR-663 overexpression suppressed PANC-1 cell invasiveness. Invasive ability of PANC-1 after transfection was assessed using Transwell assays. (*P < 0.05). **D**. eEF1A2 silencing and miR-663 overexpression induced PANC-1cell apoptosis. The apoptosis cells of PANC-1 were assessed using flow cytometry assay. (*P < 0.05). **E**. Protein level was detected by western blot assay. MMP9, pAKT and eEF1A2 were significantly reduced, and that BAD, BAX and cleaved caspase-3 were significantly increased in the miR-663 overexpressing and eEF1A2 silencing cells. β-actin was used as a reference.

To further determine the mechanisms underlying pancreatic cancer attenuation by miR-663, we focused our investigation on whether BAD, BAX, cleaved caspase-3, MMP9 and AKT were associated with the miR-663-induced attenuated proliferation, invasion and pro-apoptotic. As shown in Figure 9E, together with their protein abundances, MMP9, pAKT and eEF1A2 were significantly reduced in the PANC-1 cells overexpressing miR-663 and in the PANC-1 cells with silenced eEF1A2, as compared to control ones. BAD, BAX and cleaved caspase-3 were significantly increased in the PANC-1 cells overexpressing miR-663 and PANC-1 cells with silenced eEF1A2. According to these results, we found that the knockdown of eEF1A2 and the overexpression of miR-663 result in similar biological effect on pancreatic cancer cells, and that the attenuation is more evident in PANC-1 cells overexpressing miR-663. The result revealed that the attenuation effect of miR-663 on pancreatic cancer occurs at least partially by targeting eEF1A2; at the same time, there were other targets taking part in the process. The study demonstrated that miR-663 can act as a potential target for the treatment of pancreatic cancer in the future.

## Discussion

miR-663 is expressed in Homo sapiens and Pan troglodytes. miR-663 belongs to the primate-specific miRNAs that possibly attribute to the vertebrates’ evolution, development, and carcinogenesis [31-34]. The effect of miR-663 in malignant progression is controversial, because it could act as a tumor attenuate molecular or promoter in an organ-specific fashion [6,7]. The clinical relevance of miR-663 in pancreatic cancer remains unknown. Our present study represents the first comprehensive analysis of miR-663 in pancreatic cancer. We selected miR-663 as the target molecule from miRNA profiling, and then identified miR-663 as a tumor attenuate molecular that can attenuate the proliferation and invasion of pancreatic cancer. Mechanistically, we identified eEF1A2 as a direct and functional target of miR-663, which deepened our understanding of the mechanisms underlying pancreatic cancer progression.

Our study has demonstrated that eEF1A2 is significantly upregulated and miR-663 is significantly downregulated in pancreatic cancer. The additional results showed that eEF1A2 and miR-663 expression level were significantly associated with TNM stage and node metastasis status of the patients, but not associated with the patient’s age or gender, or with the tumor’s diameter, location or differentiation. Furthermore, while the tumor’s diameter, differentiation, clinical stage and lymph node metastasis were significantly associated with the survival of patients, the gender, age, and location were not. Since eEF1A2 and miR-663 are both associated with the survival of patient in pancreatic cancer, both may be potential biomarkers for prognosis in patients with pancreatic cancer.

Most importantly, we found that miR-663 and eEF1A2 were not only correlated inversely with each other, but were also predictive of the survival of pancreatic cancer patients. These findings highlight the potential values of miR-663 and eEF1A2 as novel prognostic biomarkers in human pancreatic cancer.

Pancreatic cancer is characterized by rapid growth and relentless invasion. Invasiveness and metastasis, the two leading causes of cancer mortalities, are especially pronounced in pancreatic cancer, which shows strikingly high invasive and metastatic potential [3]. We highlighted the therapeutic potential of miR-663 in pancreatic cancer treatment with our identification of miR-663 as a tumor attenuate molecular that attenuates the proliferation and invasion of pancreatic cancer cells both in vitro and in vivo, and that attenuates of growth and invasion of pancreatic cancer. MMPs regulate basic cellular processes including survival, migration and morphogenesis and degradation extracellular matrix during the cancer metastatic process [23]. Akt plays a key role in multiple cellular processes such as glucose metabolism, apoptosis, cell proliferation, transcription and cell migration [27]. We examined the expression levels of MMP9, Akt and pAkt(Ser473), and then found that the ectopic expression of miR-663 markedly attenuated the protein expression of MMP9, Akt and pAkt, in PANC-1 and AsPC-1 cells concomitant with the attenuation of cell invasion. These results suggest that miR-663 attenuates pancreatic cancer cell invasiveness, a property likely associated with MMP9 and Akt.

Eukaryotic elongation factor 1 alpha (eEF1A) is critical for protein synthesis because it regulates ribosomal polypeptide elongation by binding to amino-acylated tRNAs and by facilitating recruitment to the ribosome [35]. The two isoforms of eEF1A identified in humans, namely, eEF1A1 and eEF1A2, are encoded by distinct genes. eEF1A2 is a protein translation factor with important functions in tumor genesis and progression, for it is frequently overexpressed in various cancers. One recent study had demonstrated that eEF1A2 promoted cell invasion in pancreatic cancer by upregulating the expression of MMP-9 through Akt activation [22]. We identified eEF1A2 as a direct target of miR-663 by bioinformatics prediction, signal network analysis and Dual-luciferase assay. The 3′ untranslated region (3′UTR) of eEF1A2 contains a seed region for miR-663. Our pancreatic cancer tissue study has showed that eEF1A2 was significantly upregulated and miR-663 was significantly downregulated in pancreatic cancer. Most importantly, we found that miR-663 and eEF1A2 were inversely correlated with each other. These results further supported the conclusion that miR-663 targets eEF1A2.

Additionally, further study indicated that the expression of eEF1A2 could partially restore the pro-apoptotic and anti-invasion functions of miR-663. The knockdown of eEF1A2 and the overexpression of miR-663 produce similar biological effects on pancreatic cancer cells, with the effect being more obvious in PANC-1 cells overexpressing miR-663. The results revealed that the attenuation effect of miR-663 on pancreatic cancer was due at least in part to its targeting of eEF1A2, at the same time there were other targets taking part in the process. Our study has demonstrated the potential of miR-663 as a target for future pancreatic cancer treatments.

In summary, the study revealed that eEF1A2 was significantly upregulated and miR-663 was significantly downregulated in pancreatic cancer, and that both EEF1A2 and miR-663 are associated with the survival of pancreatic cancer patients. Moreover, miR-663 and eEF1A2 were correlated inversely with each other. Specifically, miR-663 attenuated the proliferation and invasion of pancreatic cells in vitro and in vivo by directly targeting eEF1A2. Most importantly, miR-663 and eEF1A2 may prove to be novel prognostic biomarkers and potential targets for future treatments of pancreatic cancer.

## Conclusions

In conclusion, we have identified that miR-663 attenuated the proliferation and invasion of pancreatic cells in vitro and in vivo by directly targeting eEF1A2. miR-663 and eEF1A2 might be potential targets for the treatment of pancreatic cancer in the future.

## Materials and methods

### Patients and tissue specimens

The tissue specimens were collected from 68 patients with pancreatic cancer who had undergone either pancreaticoduodenectomy or distal pancreatectomy between 2007 and 2009 at the First Affiliated Hospital of Zhengzhou University and the Henan Tumor Hospital of Zhengzhou University in Zhengzhou, China.

After the frozen specimens were HE stained and examined for clinicopathological features by surgical pathologists, they were then snap frozen in liquid nitrogen. Normal pancreas tissues adjacent to tumors were used as controls. None of the cancer patients in this study had received preoperative radiation or chemotherapy. Informed consent was obtained from the patients. The clinicopathologic features of these patients have been summarized in Table 1. The 68 patients with complete information were followed up after operation until February 1st, 2014, with a median follow-up time of 17.8 months. The study was approved by the Research Ethics Committee of Zhengzhou University.

### Cell culture

Human pancreatic cell line HPDE6-C7 and pancreatic cancer cell lines PANC-1, Capan-2, SW1990, BxPC3 and AsPC-1 were purchased from the Type Culture Collection of the Chinese Academy of Sciences (Shanghai, China). Subsequently, these cell lines were cultured in RPMI-1640 medium supplemented with 10% fetal bovine serum (FBS, Gibco, Australia), 100 U/ml penicillin, and 50 μg/ml streptomycin in incubators with humidified atmosphere of 5% CO_2_ and 95% air at 37°C.

### miRNA transfection

The miR-663 agomir (GMR-miR™ microRNA-663 agomir) used in this study was synthesized by Shanghai GenePharma Co. Ltd. Prior to transfection, cells were plated at a density of 1.5 × 10^5^ cells/well in 6-well plates. Once cells reached ~70% confluence, transient transfection was conducted using Lipofectamine™2000 (Invitrogen, Carlsbad, CA, USA) following the manufacturer’s instructions. Transfection efficiencies were evaluated in every experiment by qRT-PCR at 24 h post-transfection. Cells from each cell line were subdivided into three groups: the non-transfected blank group (Blank), the scrambled miR-663 transfected negative control group (NC) and the miR-663 agomir transfected group (miR-663).

### Quantitative real-time PCR

Total RNA wasextracted frompancreatic cancer tissue samples and adjacent non-tumor tissue samples using TRIzol reagent (Invitrogen, Carlsbad, CA, USA), according to the manufacturer’s instructions. 1 μg RNA was used to synthesize cDNA. And the expression levels of eEF1A2 and miR-663 were determined by qPCR (ABI 7500 fast system, Applied Biosystems, CA, USA). We used U6 small nuclear RNA (U6 snRNA) as an endogenous control for normalization. The qRT-PCR results were expressed relative to miR-663 expression levels at the threshold cycle (Ct) and were converted to fold changes (2^-ΔΔCt^).

### Western blot analysis

Total proteins of cells were extracted using RIPA buffer containing phenylme thanesulfonylfluoride (PMSF). The protein obtained was measured using a BCA Protein Assay Kit (Pierce, Rockford, IL). 30 μg of protein lysates were subjected to sodium dodecyl sulfate polyacrylamide gel electrophoresis (SDS-PAGE) and transferred onto PVDF membranes. PVDF membranes were blocked in 5% BSA in 0.05% tween 20-TBS for 1 h and incubated with primary antibody overnight at 4 diluted in foregoing blocking buffer. Dilutions for primary antibodies were as follows: anti-eEF1A2 (1:1000, Santa Cruz, USA), anti-MMP-9 (1:400, Santa Cruz, USA), anti-total Akt(1:1000, Santa Cruz, USA), anti-p-Akt (Ser 473) (1:1000, Santa Cruz, USA), anti-BAD(1:1000, Santa Cruz, USA) anti-BAX (1:1000, Santa Cruz, USA). After extensive washing with TBST, anti-rabbit IgG-HRP secondary antibody (1:5000, Santa Cruz, USA) was added. Signals were determined using a chemiluminescence detection kit (Amersham Pharmacia Biotech, Piscataway, NJ). An antibody against β-actin (Santa Cruz, USA) served as an endogenous reference.

### Cell proliferation assay

The pancreatic cancer cells were transferred to 96-wells plates at a density of 1 × 10^4^ cells/well, with five replicate wells per group. Then the relative numbers of viable cells were detected by Cell Counting Kit-8 reagents (CCK-8; Dojindo, Japan) after 0, 1, 2, 3 days of cultivation. The results were recorded using a microplate reader (Elx800; BioTek, VT, USA), in absorbance optical density at 450 nm. The experiments were independently triplicated.

### Colony formation assay

Human pancreatic cancer cell linesPANC-1 and AsPC-1 were seeded and transfected with miR-663. Cells were suspended in RPMI-1640 containing 0.35% low melting agarose, and plated onto solidified 0.6% agarose containing RPMI-1640 in six-well culture plates at a density of 1 × 10^5^ cells per dish. The plates were incubated for 2 weeks at 37 in a 5% CO_2_ incubator, and the number of colonies was counted after staining with 0.1% crystal violet solution. The colonies of more than 50 cells were manually counted. The experiments were independently triplicated.

### Transwell assay

Transwell filters (Costar, USA) were coated with matrigel (3.9 μg/μl, 60–80 μl) on the upper surface of the polycarbonic membrane (6.5 mm in diameter, 8 μm pore size). After 30 min of incubation at 37°C, the matrigel solidified and served as the extracellular matrix for tumor cell invasion analysis. Cells of the transfected and control groups (1 × 10^5^) were harvested in 100 μl of serum free RPMI-1640 medium and added to the upper compartment of the chamber. After 24 h of incubation at 37°C and 5% CO_2_, the medium was removed from the upper chamber, and then stained with methylene blue Staining Solution (Beyotime). Noninvasive cells on the upper surface were wiped with a cotton swab. The number of cells invading the matrigel was counted from three randomly selected visual fields, each from the central and peripheral portion of the filter, using an inverted microscope at 200× magnification. All experiments were performed in triplicate.

### Flow cytometry assay

Cell apoptosis was performed by flow cytometry. Human pancreatic cancer cell lines PANC-1 and AsPC-1 cells were harvested at 48 h post-transfection by trypsinization. Tumor cells were resuspended at a density of 1 × 10^6^ cells/mL in 1 × binding buffer. After double staining with FITC-Annexin V and propidium iodide (PI) using the FITC Annexin V Apoptosis Detection Kit I (BestBio, Shanghai, China), cells were analyzed using a FACScan® flow cytometer equipped with Cell Quest software (BD Biosciences, San Jose, CA, USA) according to manufacturer’s instructions to detect early and late apoptosis of cells. All experiments were performed in triplicate.

### Hoechst 33342 staining

Cells were treated with different concentrations of a1-PDX for 48 h and washed twice with cold PBS, and then incubated in the dark in 5 μL Hoechst /PI staining buffer for 15 min at 25°C. The images were recorded on a computer with a digital camera attached to the microscope, and then images were processed by the computer. The Hoechst reagent was taken up by the nuclei of the cells, and apoptotic cells exhibited a bright blue fluorescence. For quantification of Hoechst 33342 staining, the percentage of Hoechst-positive nuclei per optical field (at least 50 fields) was counted. All experiments were performed in triplicate.

### Tumor xenograft model of nude mouse

Six-week-old male nude BALB/c mice were purchased from Henan Experimental Animals Centre (Zhengzhou, China). Tumor xenograft model of nude mouse is a reliable in vivo model for tumor study. To assess the effect of miR-663 on tumorigenicity in vivo, we purchased lentivirus expressing pre-miR-663 from Shanghai GenePharma Co. Ltd and infected it into the PANC-1 cells. The 2 × 10^6^ stably transfected cells are subcutaneously injected in the dorsal scapular region of 6-week-old BALB/c nude mice (6 mice/group), which had been anesthetized by inhaling sevoflurane. The tumors formed were measured with a caliper every 7 days, and tumor volume was calculated using the following formula: volume = Л (length × width^2^)/6. Tumors were harvested after 4 weeks. These protocols were approved by the Zhengzhou University Animal Care and Use Committee.

### Dual-luciferase assay

Human eEF1A2 3′ UTR (bases108-115) fragment containing putative binding sites for miR-663 were amplified by PCR from human genomic DNA. The mutant eEF1A2 3′ UTRs was obtained by overlap extension PCR. The fragments were cloned into a pmir-GLO reporter vector (Promega), downstream of the luciferase gene, to generate the recombinant vectors pmir-GLO-eEF1A2-wt and pmir-GLO-eEF1A2-mut. For the luciferase reporter assay, PANC-1 and AsPC-1 were transiently co-transfected with miRNA (miR-633 agomir or miR-633 scramble) and reporter vectors (wild-type reporter vectors or mutant-type reporter vectors), using Lipofectamine™ 2000. Luciferase activities were measured using a Dual-Luciferase assay kit (Promega) according to manufacturer’s instructions at 48 h post-transfection.

### Statistical analyses

All statistical analyses were performed using SPSS 17.0 software. The Student *t* test or one-way ANOVA was conducted for normally distributed data. The Pearson *χ*^2^ test was used to determine the correlation between miR-663 expression and clinicopathologic features of patients. Patients’ survival was analyzed in the Kaplan-Meier method, using the log-rank test for comparison. All data represent mean ± SD. Statistical significance was set at *p* < 0.05.

## Abbreviations

eEF1A: Eukaryotic elongation factor 1-a
miR-663: microRNA-663
MMPs: Matrix metalloproteinases
PKB: Protein kinase B
